The article "Influence of Narcotrend-Assisted Anesthesia In-Depth Monitor on Cognitive Impairment of Elderly Patients under General Anesthesia" was retracted in 2023. Reasons: signs of a paper mill; compromised peer review; unreliable results or conclusions.

# Influence of Narcotrend-Assisted Anesthesia In-Depth Monitor on Cognitive Impairment of Elderly Patients under General Anesthesia

**DOI:** 10.1155/2022/2866188

**Published:** 2022-10-11

**Authors:** Maoyong Tu, Qing Zhang, Xuesheng Liu

**Affiliations:** ^1^Department of Anesthesia, The First Affiliated Hospital of Anhui Medical University, Hefei, Anhui 230022, China; ^2^Department of Anesthesia, The Second People's Hospital of Hefei, Hefei, Anhui 230011, China

## Abstract

**Objective:**

This research is designed to probe into the influence of Narcotrend- (NT-) assisted anesthesia in-depth monitor on cognitive impairment of elderly patients under general anesthesia (GA).

**Methods:**

One hundred and forty-four elderly patients with GA in our hospital from October 2020 to April 2021 were randomized into two groups, namely, NT group (supervised anesthesia under NT monitoring) and group C (anesthesia according to doctors' experience). The heart rate (HR), mean arterial pressure (MAP), and central venous pressure (CVP) were recorded before surgery (T0), at the beginning of surgery (T1), at the end of surgery (T2), and 1 day after surgery (T3). Serum of patients was obtained at these four time points for measurements of C-reactive protein (CRP), interleukin-6 (IL-6), and cortisol (Cor) levels using the enzyme-linked immunosorbent assay (ELISA). The alterations in cognitive function pre- and post-anesthesia were assessed using the mini-mental state examination (MMSE), and adverse events (AEs) during anesthesia recovery, postoperative recovery, and dosage of anesthetics were recorded.

**Results:**

At T1 and T2, MAP was higher and CVP was lower in NT group, versus group C. NT group presented higher CRP, IL-6, and Cor than group C at T1-T3. MMSE scores were higher in TN group than in group C at 12, 24, and 48 h after surgery. The incidence rates of postoperative cognitive dysfunction (POCD) and total AEs in group C were noticeably higher than those in NT group. Compared with group C, the time of anesthesia recovery, extubation, and postanesthesia care unit (PACU) residence in NT group reduced remarkably.

**Conclusions:**

NT has little effect on the physical condition of elderly patients under GA, and can reduce the dosage of narcotic drugs and promote the recovery of patients from anesthesia, which has high clinical value.

## 1. Introduction

General anesthesia (GA), combined spinal-epidural anesthesia, and inhalation anesthesia are commonly used in clinical surgical treatment at present, among which GA has the best effect and the greatest influence on patients [1]. Elderly patients are susceptible to various postoperative complications as they have relatively low tolerance to surgery and anesthesia due to poor physical quality and some comorbidities, affecting the prognosis. For example, after general anesthesia, patients may experience symptoms such as dizziness, transient memory loss, sore throat, hoarseness, and nausea and vomiting, and in severe cases, adverse complications such as deep vein thrombosis and neurological dysfunction may occur [2]. Postoperative cognitive dysfunction (POCD) is a common neurological disease after surgery, mostly seen in elderly patients [3]. It is characterized by progressive memory loss, personality changes, and postoperative cognitive loss, which will undoubtedly affect the clinical treatment effect [4]. At the present stage, the pathogenesis of POCD has not been fully elucidated. But it is shown to be closely associated with the depth of anesthesia and has been verified many times [5]. In the past, anesthesiologists usually judged the dosage of anesthesia based on the clinical signs of patients, which had great subjective influence and lacked objective and effective judgment criteria, thus leading to a higher risk of poor postoperative prognosis. Narcotrend (NT), on the other hand, is a new type of anesthesia monitoring device, which is mainly used to collect and analyze the EEG signals of patients to evaluate their anesthesia/consciousness depth [6]. Some studies believe that the use of anesthesia monitoring equipment is conducive to guiding the rational use of narcotic drugs, thereby reducing the occurrence of POCD, such as bispectral index (BIS) device-guided anesthesia which can reduce postoperative delirium and cognitive decline [7]. Other research results show that NT can reduce the dosage of anesthetics used during orthopedic surgery and promote patients to wake up earlier [8]. However, the utilization rate of NT in China is low, and its effect is still controversial.

Accordingly, this study explored the application value of NT in elderly patients under GA, so as to provide a new method for preventing the occurrence of POCD in the future.

## 2. Materials and Methods

### 2.1. Study Population

The study participants were 144 elderly patients who underwent GA in our hospital from October 2018 to January 2020, and using the random number table method, they were grouped into NT group and group C. Inclusion criteria included patients aged ≥60 and met the indications of surgical treatment under GA, with the American Society of Anesthesiologists (ASA) Grade I-II [9], and consent form signed by the patients themselves or their next of kins. The exclusion criteria included intolerance to GA or allergy to narcotic drugs, presence of consciousness disturbance before operation or mental illness, and use of drugs affecting central nervous system function within three months before operation. In addition, patients complicated with severe diseases of the vital organs such as heart, liver, kidney, and lung were excluded as well as those transferred to intensive care unit (ICU) after surgery. This study was approved by the internal Medical Ethics Committee.

### 2.2. Anesthesia Intervention

The patient's physical condition was first assessed as soon as he/she was admitted to our hospital. After entering the operating room, the venous channel was established routinely, and the liquid was replenished at a dose of 10 mL/kg per hour. The arterial pressure was measured by puncture of the radial artery, and vital signs such as electrocardiogram, heart rate (HR), and pulse oxygen saturation were monitored. After removing the grease between the patient's forehead and eyebrows with cotton balls, Narcotrend (Chindex Medical Limited, China) electrodes were placed in the above mentioned area with a distance greater than 8 cm and the resistance less than 6 K*Ω*. The Narcotrends were then connected to the power source to collect anesthesia data from the patient. Both groups of patients underwent intratracheal intravenous combined anesthesia.

The methods of anesthesia induction were intravenous injection of midazolam (Jiangsu Nhwa Pharmaceutical Co., Ltd., H20143222) and sufentanil (Jiangsu Enhua Pharmaceutical Co., Ltd., H20143315) at 0.05-0.1 mg/kg and 0.3-0.4 *μ*g/kg, respectively, as well as targeted infusion of propofol (Hebei Yipin Pharmaceutical Co., Ltd., H20093542). The concentration of narcotics was controlled at 2.0 *μ*g/mL initially and was gradually increased and reasonably adjusted according to the patient's condition. After coma, 0.6-0.8 mg/kg rocuronium (Zhejiang Xianju Pharmaceutical Co., Ltd., H20090070) was intravenously injected into the patient. When the patient's muscles relaxed and began to recover, breathing control was conducted using the anesthesia machine with the air-assisted tidal volume controlled at 8-10 mL/kg, the breathing frequency at 12 beats/min, the breathing ratio at 1 : 2, and the end-tidal carbon dioxide partial pressure (PetCO_2_) within 35-45 mmHg. After successful GA, the NT group was assessed with reference to the NT monitor data to evaluate the depth of anesthesia, based on which the anesthetic dose was adjusted to control the anesthesia depth in the range of D2-E1. In group C, the depth of anesthesia was determined according to the clinical experience of anesthesiologists. In the process of judgment, the clinical manifestations of patients were closely observed to maximize the accuracy of the evaluation results. Intraoperatively, target-controlled infusion of propofol, and intermittent intravenous infusion of sufentanil and cisatracurium were performed based on the patient's condition, and the concentration of propofol was reasonably controlled according to the course of surgical treatment to ensure the depth of anesthesia and avoid excessive anesthesia. Propofol infusion was stopped when suturing the skin. Postoperatively, patient-controlled analgesia was carried out with analgesia pump. The types and doses of analgesics were sufentanil (100 *μ*g), butorphanol (4 mg), and the total dose of analgesic solution was 150 mL. Postoperative analgesia, as the standard practice of this department, depends on the type and duration of operation. None of the subjects received anesthetic antagonists during the procedure. After surgery, the patient was extubated and admitted to the postanesthesia care unit (PACU) after the spontaneous breathing was restored and the patient responded to the instructions to open the eyes (breathing >8 times/min and PetCO_2_ < 45 mmHg).

### 2.3. Outcome Measures

HR, mean arterial pressure (MAP), and central venous pressure (CVP) were recorded by Drager multiparameter ECG monitor (Dräger bedside monitor Infinity^®^ Omega-S, Shanghai Hangfei Medical Equipment Co., Ltd.) before surgery (T0), at the beginning of surgery (T1), at the end of surgery (T2), and one day after surgery (T3). Venous blood was collected at these four time points, and serum was obtained by centrifugation for measurements of C-reactive protein (CRP), interleukin-6 (IL-6), and cortisol (Cor) using the enzyme-linked immunosorbent assay (ELISA) strictly following the kit instructions (The kit was purchased from TransGen Biotech, China).

Cognitive function of patients was assessed using the mini-mental state examination (MMSE) [10] at 12 h before operation and 12, 24, and 48 h after the procedure. With a full score of 30 points, a score <27 indicated the presence of cognitive dysfunction, and the lower the score, the higher the degree of the disorder.

Adverse events (AEs) during anesthesia recovery and postoperative recovery were recorded. The former mainly covered restlessness, nausea and vomiting, arrhythmia, hypotension, and POCD, while the latter mainly included the time of anesthesia recovery, extubation, and PACU residence.

The nursing activities score (NAS) [11] was used to evaluate the workload of nurses since the patient entered PACU. The scale (full score: 177 points) consisted of 23 nursing items, each of which was scored according to the percentage of the time it spent in one day's working time of the nurse. The higher the score, the greater the workload.

### 2.4. Statistical Processing

Data analysis and image rendering employed SPSS 18.0 (IBM Corp, Armonk, NY, USA) and GraphPad Prism 7, respectively. Chi-square test or Fisher' s exact test was adopted to compare the counting data. The measurement data between groups were compared by independent samples *t*-test, and the means of multi-arm were compared using one-way ANOVA, followed by Dunnett-*t*-test pairwise comparison. The level of significance was taken as *P* < 0.05.

## 3. Results

### 3.1. Summary of Results

MMSE scores were higher in TN group than in group C at 12, 24, and 48 h after surgery (*P* < 0.05). The incidence rates of postoperative cognitive dysfunction (POCD) and total AEs in group C were noticeably higher than those in NT group (*P* < 0.05). Compared with group C, the time of anesthesia recovery, extubation, and postanesthesia care unit (PACU) residence in NT group reduced remarkably (*P* < 0.05).

### 3.2. Comparison of General Data

In order to ensure the reliability of the experimental results, we conducted a preliminary comparison of the clinical data of the two groups of patients before the beginning of the study. The results showed that there were no significant difference in age, body mass index (BMI), operation time, diabetes, hypertension, education level, and ASA grade between the two groups (*P* > 0.05, Table 1), indicating the comparability between the two groups of patients and feasibility for further comparison.

### 3.3. Comparison of Hemodynamic Indices

First of all, we made a preliminary comparison of hemodynamics between the two groups, and the observed indicators were HR, MAP, and CVP (Table 2). It was found that there was no significant difference in HR, MAP, and CVP between the two groups at T0 (*P* > 0.05), nor was there any significant difference in HR between groups at T1-T3 (*P* > 0.05). At T1, the MAP of group C was (92.42 ± 8.56) mmHg, and that of NT group was (85.10 ± 8.14) mmHg, both lower than that of T0, and the MAP of group C was lower than that of NT group (*P* < 0.05). At T2, MAP of both groups showed a continuous decline, and the level in group C was lower compared with NT group (*P* < 0.05). At T3, the MAP of both groups increased again, which was not different from that of T0. At T3, MAP of the two groups increased again, showing no difference with that at T0 (*P* > 0.05). As to CVP, its level increased gradually in both groups at T1 and T2, with a higher level in group C compared with NT group (*P* < 0.05). At T3, CVP of both groups decreased again to no difference from that of T0 (*P* > 0.05).

### 3.4. Comparison of Stress Response Indicators

Furthermore, the changes in stress responses were evaluated by measuring the levels of CRP, IL-6, and Cor in the two groups (Table 3). The results showed no significant differences in CRP, IL-6, and Cor between the two groups at T0 (*P* > 0.05), while significantly increased levels of these indicators in both groups at T1, with higher levels in group C compared with NT group (*P* < 0.05). At T2, CRP, IL-6, and Cor remained relatively stable in both groups, with no significant difference from those at T1 (*P* > 0.05) while higher levels in group C compared with NT group (*P* < 0.05). At T3, the levels of CRP, IL-6, and Cor in group C decreased to (399.74 ± 56.85 ng/mL), (29.26 ± 4.36 pg/mL), and (156.89 ± 22.67 ng/mL), respectively, but still higher than those in NT group (*P* < 0.05).

### 3.5. Comparison of Cognitive Function

The cognitive function of patients during treatment was assessed by the MMSE score, and the results are shown in Figure 1. The MMSE scores of group C and NT group at T0 were (29.11 ± 0.56) and (29.24 ± 0.61), respectively, showing no significant difference between the two groups (*P* > 0.05). At T1, the scores decreased to (21.76 ± 2.12) and (24.12 ± 1.65) in group C and NT group, respectively, with a lower score in group C compared with NT group (*P* < 0.05). The MMSE score showed an increase in both groups at T2, but still was lower in group C than in NT group (*P* < 0.05). At T3, the MMSE score of the two groups increased continuously, but were still lower than those at T0 (*P* < 0.05), and the score of group C was lower than that of NT group (*P* < 0.05).

### 3.6. Comparison of AEs during Anesthesia Recovery

The AEs of patients in two groups during anesthesia recovery were recorded. It was found that the AEs such as restlessness, nausea and vomiting, arrhythmia, and hypotension were not significantly different between the two groups (*P* > 0.05). However, the incidence of POCD in group C was 13.89% (10 cases), which was significantly higher than that of NT group with an incidence of only 4.17% (3 cases) (*P* < 0.05). After the final calculation of the total incidence of AEs in the two groups, it was found that the total incidence of AEs in group C was 36.11%, which was also higher than that in NT group (12.50%) (*P* < 0.05, Table 4).

### 3.7. Comparison of Postoperative Recovery and NAS Scores

Postoperative recovery of patients in the two groups was recorded. It was found that the time of anesthesia recovery, extubation, and PACU residence were significantly shorter in NT group compared to group C (*P* < 0.05). The postoperative recovery of the two groups of patients was further evaluated by the NAS score. The results showed that the NAS score of group C was (34.42 ± 9.85), while that of NT group was (30.65 ± 9.72), with statistical significance between the two groups (*P* < 0.05, Table 5).

## 4. Discussion

GA is a common anesthesia method in surgery. Today, patients' anesthesia depth is mainly evaluated by the changes of basic indices such as HR and blood pressure, but these indices fluctuate widely due to the influence of personal physical state and psychological state [12]. Besides, the risk of anesthesia in elderly patients is significantly higher than that in young patients due to the decline of physical function and frequent complication of cardiovascular and cerebrovascular diseases [13]. Accordingly, it is necessary to choose an ideal mode of anesthesia.

NT is a new EEG/consciousness depth monitoring system, which can collect and analyze the instant EEG signals of patients' brains through ECG electrodes [14]. NT can subdivide the original EEG into six stages, namely, A (awake), B0-B2 (sedation), C0-C2 (shallow anesthesia), D0-D2 (routine anesthesia), E0-E2 (deep anesthesia), and F0-F2 (burst suppression), among which D1-D2 is the best for GA induction. A number of previous clinical studies have indicated that NT can achieve the best anesthetic effect with less anesthetics and shorten the recovery time of patients [15]. Our research identified notably shortened time of recovery, extubation, and PACU residence in NT group, which agreed with the preceding research results. As we all know, PACU nursing is an important link in accelerating rehabilitation surgery. Therefore, we evaluated the impact of TN on the workload nurses in PACU. The results revealed statistically lower NAS scores in NT group compared with group C, indicating that TN can reduce the workload of nurses in PACU, which may be related to the fact that TN can shorten the anesthesia recovery time of patients.

Characterized by inability to concentrate, memory loss, confusion of thinking and listlessness, POCD refers to the long-term cognitive dysfunction of patients after surgery, which will not only prolong the hospitalization time, but also have an adverse impact on the postoperative rehabilitation of patients [16, 17]. Hence, reducing the occurrence of POCD is an important topic for clinicians. It was found in this study that in comparison with group C, the MMSE scores were higher in TN group at 12, 24, and 48 h after surgery, and the incidence of POCD was lower, indicating that NT has less influence on the neurological function of elderly patients under GA.

Tissue trauma, pain perception, and psychological emotion will activate hypothalamus-pituitary-adrenal axis and sympathetic nervous system, triggering stress response, thereby reducing the perioperative stress response of patients, which is conducive to patients' recovery and can reduce the occurrence of potential complications [18, 19]. Evidence has shown that appropriate depth of anesthesia can reduce the stress response of patients undergoing surgery and improve the hemodynamic stability of patients [20, 21]. The results of this study revealed that at T1 and T2, the MAP value was higher and the CVP value was lower in NT group compared with group C, and higher CRP, IL-6, and Cor were determined in NT group at T1-T3. It indicates that NT can reduce the influence of GA on the physical condition of elderly patients. The functions of various tissues and organs of patients are in an unstable state during the anesthesia recovery after GA, coupled with the intraoperative use of muscle relaxants, anesthetic residues, and the incomplete recovery of the body's protective reflex, resulting in the susceptibility to complications such as arrhythmia and POCD, which is detrimental to the postoperative outcomes of patients [22, 23]. Furthermore, this study made statistics on AEs during anesthesia recovery and found a notably lower incidence rate in NT group. The reason is that NT can judge the depth of anesthesia through monitoring indicators, so as to adjust the dosage and injection speed of intravenous anesthetics, improve the anesthetic effect, and make the patient's body less affected by surgery and narcotic drugs.

Of course, this study also has many limitations that need to be improved. For example, there are some other anesthesia methods currently in clinical practice, and it is worthwhile to conduct research and analyze the application value of NT in other anesthesia methods. Second, for different types of operations, the doses of anesthesia drugs are different, which also requires us to conduct more detailed classification and comparison. Finally, the number of subjects in this study is small, and there may be statistical randomness, and we should extend the follow-up time of patients to further evaluate the application value of NT.

## 5. Conclusion

NT has little influence on the physical condition of elderly patients under GA and can reduce the dosage of narcotic drugs and promote patients to wake up earlier, which has high clinical application value.

## Figures and Tables

**Figure 1:** Cognitive function comparison. Note: ^∗^*P* < 0.05 vs group C, ^#^*P* < 0.05 vs 12 h before surgery, ^&^*P* < 0.05 vs 12 h after operation, ^@^*P* < 0.05 vs 24 h after operation.

**Table 1:** Comparison of general data between two groups ([*n*(%)], $\bar{x}\pm s$).

	Group C (*n* = 72)	NT group (*n* = 72)	*χ* ^2^/*t*	*P*
Gender			0.457	0.499
Female	32 (44.44)	28 (38.89)		
Male	40 (55.56)	44 (61.11)		
Age	69.25 ± 7.58	70.89 ± 8.08	1.256	0.211
BMI (kg/cm^2^)	23.63 ± 2.25	23.34 ± 2.43	0.743	0.459
Operation time (min)	148.25 ± 18.47	145.77 ± 20.15	0.770	0.443
Diabetes			0.538	0.463
Have	23 (31.94)	19 (26.39)		
No	49 (68.06)	53 (73.61)		
Hypertension			0.123	0.726
Have	24 (33.33)	26 (36.11)		
No	48 (66.67)	46 (63.89)		
Education			1.150	0.284
>Junior high	26 (36.11)	20 (27.78)		
≤Junior high school	46 (63.89)	52 (72.22)		
ASA rating			0.265	0.607
I	29 (40.28)	26 (36.11)		
II	43 (59.72)	46 (63.89)		

**Table 2:** Comparison of adverse events during anesthesia recovery [*n* (%)].

	Group C (*n* = 72)	NT group (*n* = 72)	*χ* ^2^	*P*
Restlessness	5 (6.94)	2 (2.78)	1.351	0.245
Feel sick and vomit	7 (9.72)	3 (4.17)	1.719	0.190
Arrhythmia	2 (2.78)	1 (1.39)	0.340	0.560
Low blood pressure	2 (2.78)	0 (0.00)	2.028	0.154
POCD	10 (13.89)	3 (4.17)	4.143	0.042
Total incidence	26 (36.11)	9 (12.50)	10.909	0.001

**Table 3:** Comparison of hemodynamic indices $\left(\bar{\chi }\pm s\right)$.

	Group C (*n* = 72)	NT group (*n* = 72)	*t*	*P*
HR (times/min)				
T0	82.56 ± 8.65	84.12 ± 9.12	1.053	0.294
T1	80.29 ± 9.01	82.75 ± 8.65	1.671	0.097
T2	80.24 ± 6.82	82.05 ± 6.87	1.587	0.115
T3	81.56 ± 7.83	83.00 ± 6.59	1.194	0.235
MAP (mmHg)				
T0	92.42 ± 8.56	93.26 ± 9.24	0.566	0.572
T1	76.23 ± 8.23^∗^	82.10 ± 8.14^∗^	4.303	<0.001
T2	77.14 ± 8.49^∗^^#^	83.10 ± 8.66^∗^^#^	2.989	0.004
T3	91.56 ± 7.62^#@^	92.12 ± 7.21^#@^	1.262	0.209
CVP (H2O)				
T0	6.26 ± 1.14	6.38 ± 1.02	0.666	0.507
T1	8.63 ± 1.01^∗^	7.83 ± 1.11^∗^	4.523	<0.001
T2	8.13 ± 1.04^∗^^#^	7.12 ± 1.04^∗^^#^	5.827	<0.001
T3	6.77 ± 1.16^#@^	6.58 ± 0.95^#@^	1.075	0.284

Note: ^∗^*P* < 0.05 vs group C, ^#^*P* < 0.05 vs 12 h before surgery, ^&^*P* < 0.05 vs 12 h after operation, ^@^*P* < 0.05 vs 24 h after operation.

**Table 4:** Comparison of stress response indicators.

	Group C (*n* = 72)	NT group (*n* = 72)	*t*	*P*
CRP (ng/mL)				
T0	322.55 ± 56.35	320.16 ± 55.67	0.256	0.798
T1	466.78 ± 52.75^∗^	402.47 ± 48.28^∗^	7.631	<0.001
T2	452.24 ± 47.36^∗^^#^	398.75 ± 48.57^∗^^#^	6.691	<0.001
T3	399.74 ± 56.85^∗^^#@^	359.79 ± 50.95^∗^^#@^	4.440	<0.001
IL-6 (pg/mL)				
T0	15.47 ± 3.89	16.02 ± 3.67	0.873	0.384
T1	36.36 ± 5.87^∗^	29.47 ± 5.77^∗^	7.121	<0.001
T2	40.25 ± 5.54^∗^^#^	28.86 ± 5.53^∗^^#^	12.350	<0.001
T3	29.26 ± 4.36^∗^^#@^	23.36 ± 4.67^∗^^#@^	7.836	<0.001
Cor (ng/mL)				
T0	127.25 ± 18.74	125.71 ± 17.17	0.514	0.608
T1	163.74 ± 27.67^∗^	152.14 ± 20.53^∗^	2.857	0.005
T2	178.25 ± 25.36^∗^^#^	155.75 ± 22.65^∗^^#^	5.615	<0.001
T3	156.89 ± 22.67^∗^^#@^	142.61 ± 26.73^∗^^#@^	3.457	<0.001

Note: ^∗^*P* < 0.05 vs group C, ^#^*P* < 0.05 vs 12 h before surgery, ^&^*P* < 0.05 vs 12 h after operation, ^@^*P* < 0.05 vs 24 h after operation.

**Table 5:** Comparison of postoperative recovery and NAS scores ($\bar{\chi }\pm s$).

	Group C (*n* = 72)	NT group (*n* = 72)	*t*	*P*
Wake up time (min)	15.35 ± 4.25	12.67 ± 4.67	3.601	<0.001
Extubation time (min)	23.14 ± 5.17	19.36 ± 4.81	4.542	<0.001
PACU stay time (min)	48.64 ± 10.69	43.56 ± 9.84	2.967	0.004
NAS score (points)	34.42 ± 9.85	30.65 ± 9.72	2.312	0.022

## Data Availability

The datasets used and/or analyzed during the current study are available from the corresponding author on reasonable request.
